# A Study on the Role of Intelligent Medical Simulation Systems in Teaching First Aid Competence in Anesthesiology

This article has been retracted.

**DOI:** 10.1155/2022/8163546

**Published:** 2022-04-21

**Authors:** Wei He, Jiayu Lu, Wei Zheng, Xingyu Zhang, Zhaoxiang Yu, Lin Shen, Duo Zhang

**Affiliations:** ^1^Department of Anesthesiology, The Affiliated Hospital of Beihua University, Jilin City, Jilin Province 132000, China; ^2^The Affiliated Hospital of Beihua University, Jilin City, Jilin Province 132000, China

## Abstract

Anesthesiology is a subject with strong practicality and application. Undergraduate anesthesiology teaching needs to strike a balance between theoretical knowledge, clinical skill training, and clinical thinking development. Clinical probation and practice are an important part of undergraduate anesthesia teaching. Traditional clinical teaching uses real patients for demonstration and training, but as patients become more self-protective and less cooperative, there are not enough patients for clinical skill training. Simulation is to teach medical scenes in real life under the control of standardized technical guidelines and parameters. Since then, with the rapid development of computer technology, simulation technology and simulation teaching have been greatly developed and are more and more used in clinical teaching, skill evaluation, and scientific research. This study explores the effective methods of clinical teaching in anesthesiology by comparing the effectiveness of traditional teaching methods and simulation teaching methods in undergraduate clinical teaching. It is difficult to combine theory and practice in first aid, which does not allow them to directly receive and deal with emergency medical treatment and resuscitation. In China's current medical environment and patients' high demand for medical services, it is imperative to vigorously carry out simulated medical education. In the eastern part of Inner Mongolia, according to the advantages of teaching hospitals, our hospital took the lead in carrying out the simulation education project, which is still in the exploratory stage and not systematic enough. This study will help us to better carry out simulation teaching and improve the clinical skills of medical students in the future. *Methods*. The student group and class took the advanced simulator training as the experimental group, applied the advanced integrated simulator and other systems of the Norwegian company, referred to the international guidelines for cardiopulmonary resuscitation and cardiovascular first aid in 2005, and practiced in the emergency department during the clinical internship and “emergency clinical simulation training” course. The course includes basic life support, advanced life support, and comprehensive training of CPR (cardiopulmonary resuscitation) and endotracheal intubation. *Results*. The passing rate of simulated first aid practice was 94.4%; 100% of the students think it is necessary to set up the course, 91% of the students think it is practical, 91% of the students think the course content is reasonable and perfect, and 77%–100% of the students think the course has improved their first aid operation ability, comprehensive application of knowledge, and clinical thinking ability. *Conclusion*. Carrying out the course of “clinical simulated first aid training” through the advanced simulator system can effectively improve the interns' clinical first aid operation ability, teamwork ability, and self-confidence, improve the students' clinical thinking and judgment ability, and improve the service level to patients.

## 1. Introduction

Medical simulation is a branch of simulation technology, which is used for education, training, and research on various topics in the medical field. Medical simulation education is an educational method that uses simulation technology to replace real patients and create simulated patients and simulated clinical scenes for clinical teaching and practice [1]. The purpose of using simulation equipment (various local functional models, interactive computer models, and simulation systems, such as virtual technology) instead of real-time Spanish is to find solutions to meet the training challenges of medical students in the clinical stage of basic skills [2]. The application of high-end simulation technology in medical education, especially in the field of emergency medicine with the same high risk, has only been more than a decade. As early as the 1990s, some Western countries with advanced medical practice suggested changing the traditional mode of medical education, such as the General Medical Council (GMC), which issued a proposal to reform medical education, combining theoretical medical knowledge, patient communication skills, and clinical skills training [3]. The GMC has issued a proposal to reform medical education, combining theoretical knowledge, communication skills, and clinical skills. Therefore, clinical skill laboratories and medical simulation education centers of various scales have been established, and a number of medical simulators have been gradually used in clinical teaching. In 1996, the Loreal Aerospace Research Center (USA) founded the medical education technology company (MET) to develop a complex medical simulation teaching system, namely, the human patient simulator (HPS). The system uses advanced computer technology to simulate real human pathology and various clinical cases and treatment scenes, organ functions, and various human systems through skin contact. It has multimedia technology, physiological data display and monitoring, computer technology programming, recording, and storage [4]. The University of Bristol in the United Kingdom has established a relatively mature simulation education research center. The Universities of Hong Kong, Sydney, Australia, Fordham, and Canada have also established simulation centers. In 2006, Beijing Xuanwu Hospital established an endourological simulation center, and simulation education centers also appeared in the Southwest Hospital, Ningbo Health School, Chaoyang Hospital, and other areas, starting a systematic medical simulation education [5]. In order to improve the level of clinical skill training and medical simulation education in China, give full play to the characteristics and advantages of medical simulation education and quickly improve the clinical skills of medical staff, and the Career Development Department of the Chinese Medical Association held the “first advanced seminar on clinical skill training and medical simulation education” in the Chongqing Southwest Hospital in January 2008. By 2009, more than 400 medical schools in China had established simulation centers to provide simulation education [6]. In view of the contradiction between China's current medical environment and patients' high demand for medical services, it is imperative to vigorously develop simulated medical education [7].

The development of modern medicine has made emergency medicine an independent medical discipline. Emergency medicine has become one of the important symbols reflecting the level of clinical medical science [8]. It is important to train medical personnel who are suitable for the needs of China's medical service system and have solid basic skills in emergency medicine and first aid. First aid is highly practical, highly acute, rapidly changing, and complex [9–12]. The emergence of medical simulation products can solve this problem to a large extent and will play a very important role in the training of basic clinical skills, especially in the training of emergency medical techniques. The integrated simulator realistically simulates various pathological and physiological changes, expresses various clinical symptoms and signs, can be set up at any time according to clinical teaching needs, does not involve doctor-patient disputes, does not cause harm to patients, and can be used to teach [13]. Anesthesia simulator anesthesia simulation software can simulate patients, anesthesia machines, and monitors in the software interface. Users can check patients, control airways, implement ventilation, administration, and rehydration through mouse control and a simple menu. The software includes 80 patients, covering various anesthesia scenes, including general anesthesia, local anesthesia, cardiac, neurosurgical, pediatric, and obstetric anesthesia. More than 100 kinds of drug reactions are built in. The cardiovascular system, respiratory system, and pharmacological parameters can change to varying degrees, showing normal and different degrees of disease states. It can also simulate complex pathophysiological processes and critical events, such as malignant hyperthermia. The automatic recording system stores all diagnostic and treatment inputs, allows the independent management of cases without instructors, and automatically summarizes the evaluation. In addition, the real-time consultation system can provide management suggestions at any time during training.

The application of simulation systems is of great significance to cultivate medical students' clinical practical ability, clinical comprehensive diagnosis and treatment ability, and team cooperation ability [14]. In the eastern part of Inner Mongolia, our college took the lead in carrying out the simulation education course. At present, it is still in the exploratory stage and not systematic enough. This study is to accumulate experience, better carry out medical simulation education in the future, and improve the clinical skills of medical students in our hospital. In this experiment, the “clinical simulated first aid training” course conducted through the advanced simulation system can effectively improve the interns' clinical first aid operation ability, teamwork ability, and self-confidence, as well as the students' clinical thinking and judgment ability, so as to improve the service level for patients [15].

## 2. Materials and Methods

### 2.1. Information

A total of 102 trainees and clinical postgraduate students from the department of respiratory medicine in 2021 were divided into two groups by batch. There were 42 males and 60 females, with a mean age of 24.3 years. There was no statistically significant difference between the two groups in terms of age, gender, admission score, and examination results of undergraduate courses (*P* > 0.05).

## 3. Methods

The 102 inpatient interns and clinical master students were divided into two groups according to batches. Control group: 52 students were trained in respiratory medicine according to the traditional clinical teaching plan. Experimental group: 50 students received the training of traditional clinical teaching plan in respiratory medicine. After entering respiratory medicine, they used an intelligent medical simulation system for teaching. The intelligent medical simulation system is arranged during normal working hours to ensure that there is no difference in learning time between the two groups. The teaching objectives include anesthesia, cardiopulmonary resuscitation, mechanical ventilation, endotracheal intubation, tracheotomy, annular nail puncture, sputum suction, arterial blood collection and arterial blood gas analysis, thoracic puncture and other punctures, cardiopulmonary and abdominal examination, ECG (electrocardiogram) operation and analysis, medical record analysis, and other basic skills. After completing the learning objectives, evaluate the two groups of students. A questionnaire survey was conducted on the teaching methods of the two groups of students and the learning methods of the experimental group of the intelligent medical comprehensive simulation system.

### 3.1. Statistical Analysis

The data were statistically analyzed using SPSS (Statistic Package for Social Science) 15.0 software, and the measurement data were expressed as (mean ± standard deviation) using the *t*-test.

## 4. Results

### 4.1. Comparison of Examination Results

The theoretical knowledge, clinical skills, and general ability were assessed for both groups, as given in Table 1. The participants in the experimental group gave feedback on the learning method of the intelligent medical simulation system, as given in Table 2. 94.0% of the participants in the experimental group and 53.8% of the participants in the control group gave feedback on their satisfaction with the teaching method, with a high statistical significance (*P* < 0.01), as given in Table 3.

## 5. Discussion

### 5.1. The Advantages of Teaching with an Intelligent Integrated Medical Simulation System

Traditional medicine is based on knowledge inculcation and pays insufficient attention to clinical skill teaching, which makes it difficult to meet the requirements of clinical professional posts, resulting in students' low interest in learning, poor mastery of theoretical knowledge, poor practical ability, and the separation of “learning” and “use” [16]. In the teaching of respiratory first aid, the intelligent medical comprehensive simulation system is applied to simulate the real clinical situation, simulate the disease and pathophysiological changes of patients, start with the basic knowledge of respiratory pathology, guide students to master clinical theoretical knowledge and operation skills, improve students' adaptability and sense of cooperation, and achieve the purpose of mastering theoretical knowledge and applying theoretical knowledge to clinic [17].

This experiment uses an intelligent medical comprehensive simulation system for clinical teaching and explores a new method of respiratory first aid teaching. The results show that compared with the control group, the theoretical test, clinical skill test, and comprehensive ability evaluation of the experimental group are highly statistically significant [18]. This is because the intelligent medical integrated simulation system stimulates students' learning initiative and strong learning interest. The simulation system simulates the real clinical environment, making it easier for students to understand the theoretical knowledge, so as to make the theoretical knowledge more profound and firm [19]. The results of a student questionnaire survey show that the training of the intelligent medical comprehensive simulation system stimulates students' interest in learning, helps to deepen their understanding and memory of theoretical knowledge, and improves their practical operation ability, adaptability, judgment ability, and teamwork ability. It has become a teaching method loved by most students, and most of them hope to adopt this teaching method more in the future [20].

### 5.2. Shortcomings in the Teaching of Intelligent Medical Integrated Simulation Systems

There is still a gap between the intelligent medical integrated simulation system and the actual clinical environment, and most of the clinical cases designed are typical cases, which may cause students' perceptions to be biased, as the actual occurrence of cases in the clinic is affected by many factors and the clinical situation is highly variable. It is more difficult to complete face-to-face doctor-patient communication training in the teaching of intelligent medical integrated simulation systems. Due to human body differences, simulated patients cannot completely replace real people as clinical training objects nor can simulated instruments simulate certain complex emergencies that occur in real environments. It is necessary to combine the teaching of the intelligent medical integrated simulation system with traditional clinical teaching, so as to achieve twice the result with half the effort [21, 22].

In conclusion, intelligent medical integrated simulation system teaching solves the problem of poor practical ability of medical students due to the lack of clinical practice opportunities and is an important and effective supplement to traditional clinical teaching methods, as well as a bridge to apply theoretical and practical knowledge to clinical practice. By reasonably integrating intelligent medical simulation system teaching into the traditional clinical teaching process, it can deepen medical students' understanding and application of theoretical knowledge, improve their clinical practice ability, and cultivate more practical clinical talents.

## 6. Conclusions

Foreign research on simulation education is relatively mature. In our hospital, we took the lead in developing the simulation education project according to the advantages of the teaching hospital. The project is still in the exploratory stage and not systematic enough. This study has accumulated preliminary experience for better carrying out medical simulation education and improving the first aid skills of medical students in our hospital in the future. Through the training of advanced intelligent simulator systems, students' mastery of theoretical knowledge of first aid, practical operation ability, and clinical cooperation ability have been significantly improved. Students can accept the application of the advanced intelligent simulation system in teaching, and the teaching effect is significantly improved.

## Figures and Tables

**Table 1:** Comparison of the examination results of the two groups of students.

Assessment items	Experimental group (*n* = 50)	Control group (*n* = 52)	*t*	*P*
Theoretical assessment	85.2±8.2	76.9±5.3	11.42	<0.01
Skill assessment	88.5±6.5	67.7±4.5	24.13	<0.01
Comprehensive ability assessment	87.6±7.2	73.1±4.1	17.25	<0.01

**Table 2:** Participants' feedback on the intelligent medical integrated simulation system course questionnaire.

Evaluation items	Student feedback		
Improve learning enthusiasm and interest	Helpful 100% (50/50)	General 0% (0/50)	No help 0% (0/50)
Influence on clinical thinking	Helpful 90% (45/50)	General 10% (5/50)	No help 0% (0/50)
Deepen the understanding and mastery of knowledge	Helpful 96% (48/50)	General 4% (2/50)	No help 0% (0/50)
Practical operation ability	Increased by 100% (50/50)	Slightly increased by 0% (0/50)	No increase of 0% (0/50)
Teamwork ability	Increased by 80% (40/50)	Slightly increased by 20%	No increase of 0% (0/50)
Doctor-patient communication skills	Increased by 30% (15/50)	Slightly increased by 20% (10/50)	No increase of 50% (25/50)
Adaptability and judgment	Increased by 92% (46/50)	Slightly increased by 8% (4/50)	No increase of 0% (0/50)
Problem solving ability	Increased by 92% (46/50)	Slightly increased by 8% (4/50)	No increase of 0% (0/50)
Necessity of offering this course	Necessary 100% (50/50)	Slightly increased by 6% (3/50)	No increase of 0% (0/50)
Practicality of the course	Significant effect 100% (50/50)	Unnecessary 0% (0/50)	It does not matter 0% (0/50)
Satisfaction with the course	Very satisfied 100% (50/50)	Also 0% (0/50)	Dissatisfied 0% (0/50)
Course content	Reasonable improvement 84% (42/50)	Need to add 10% (5/50)	Content to be deleted 6% (3/50)

**Table 3:** Results of questionnaire feedback on student satisfaction with teaching methods in both groups.

Group	*n*	Satisfied	Dissatisfied	Indifferent	Satisfaction rate (%)	*t* value	*P*
Experience group	50	47	1	2	94	14.98	<0.01
Control group	52	28	20	4	53.8	-	-

## Data Availability

The datasets used in this study are available from the corresponding author upon request.

## References

[1] McKendrick M., Yang S., McLeod G. A. (2021). The use of artificial intelligence and robotics in regional anaesthesia. *Anaesthesia*.

[2] Benkhedda S., Bendella F. (2019). FASim: a 3D serious game for the first aid emergency. *Simulation & Gaming*.

[3] Martinelli S. M., Isaak R. S., Schell R. M., Mitchell J. D., McEvoy M. D., Chen F. (2019). Learners and ltc. *Anesthesiology*.

[4] Friedl K. E., O’Neil H. F. (2013). Designing and using computer simulations in medical education and training: an introduction. *Military Medicine*.

[5] Haber J. A., Ellaway R. H., Chun R., Lockyer J. M. (2017). Exploring anesthesiologists’ understanding of situational awareness: a qualitative study. *Canadian Journal of Anesthesia/Journal canadien d’anesthésie*.

[6] Radhakrishnan B., Katikar M. D., Myatra S. N., Gautam P. L., Vinayagam S., Saroa R. (2022). Importance of non-technical skills in anaesthesia education. *Indian Journal of Anaesthesia*.

[7] Jones C. P. L., Fawker-Corbett J., Groom P., Morton B., Lister C., Mercer S. J. (2018). Human factors in preventing complications in anaesthesia: a systematic review. *Anaesthesia*.

[8] Bowness J., El‐Boghdadly K., Burckett‐St Laurent D. (2021). Artificial intelligence for image interpretation in ultrasound‐guided regional anaesthesia. *Anaesthesia*.

[9] Wang N., Han W., Wang R., Wang J. (2019). The application of intelligent simulated human teaching equipment in clinical practice. *IOP conference series: materials science and engineering*.

[10] Prineas S., Cuyx L., Smet J. (2021). e-Learning in regional anesthesia. *Current Opinion in Anaesthesiology*.

[11] Chernikova O., Heitzmann N., Stadler M., Holzberger D., Seidel T., Fischer F. (2020). Simulation-based learning in higher education: a meta-analysis. *Review of Educational Research*.

[12] Li J., Zhou Z., Li J. (2019). Decentralized on-demand energy supply for blockchain in Internet of Things: a microgrids approach. *IEEE transactions on computational social systems*.

[13] Epstein J. H., Levin M., Jowell M. S. Agent based simulation for training and assessing students in the field of anesthesiology.

[14] Cote C. D., Kim P. J. (2019). Artificial intelligence in anesthesiology: moving into the future. *University of Toronto Medical Journal*.

[15] Haskins S. C., Bronshteyn Y., Perlas A. (2021). American Society of Regional Anesthesia and Pain Medicine expert panel recommendations on point-of-care ultrasound education and training for regional anesthesiologists and pain physicians-part I: clinical indications. *Regional Anesthesia and Pain Medicine*.

[16] Komorowski M., Fleming S., Mawkin M., Hinkelbein J. (2018). Anaesthesia in austere environments: literature review and considerations for future space exploration missions. *NPJ microgravity*.

[17] Kassahun Y., Yu B., Tibebu A. T. (2016). Surgical robotics beyond enhanced dexterity instrumentation: a survey of machine learning techniques and their role in intelligent and autonomous surgical actions. *International Journal of Computer Assisted Radiology and Surgery*.

[18] McAlpin E., Bergner Y., Levine M. (2021). Summative assessments of web. *European Journal of Dental Education*.

[19] Wang N., Yu J., Wang L., Hao X. (2020). Application of intelligent control in medical education. *Data Processing Techniques and Applications for Cyber-Physical Systems (DPTA 2019)*.

[20] Zhang Z.-wan, Wu Di, Zhang C.-jiong (2021). Study of cellular traffic prediction based on multi-channel sparse LSTM. *Computer Science*.

[21] Ramsingh D., Bronshteyn Y. S., Haskins S., Zimmerman J. (2020). Perioperative point-of-care ultrasound. *Anesthesiology*.

[22] Jin Q., Jiang X., Park J., Li S. (2014). *Frontier and Future Development of Information Technology in Medicine and Education*.

